RETRACTED

# Measures of Clade Confidence Do Not Correlate with Accuracy of Phylogenetic Trees

**DOI:** 10.1371/journal.pcbi.0030051

**Published:** 2007-03-16

**Authors:** Barry G Hall, Stephen J Salipante

**Affiliations:** 1 Bellingham Research Institute, Bellingham, Washington, United States of America; 2 Department of Genome Sciences, University of Washington, Seattle, Washington, United States of America; University of Chicago, United States of America

## Abstract

Metrics of phylogenetic tree reliability, such as parametric bootstrap percentages or Bayesian posterior probabilities, represent internal measures of the topological reproducibility of a phylogenetic tree, while the recently introduced aLRT (approximate likelihood ratio test) assesses the likelihood that a branch exists on a maximum-likelihood tree. Although those values are often equated with phylogenetic tree accuracy, they do not necessarily estimate how well a reconstructed phylogeny represents cladistic relationships that actually exist in nature. The authors have therefore attempted to quantify how well bootstrap percentages, posterior probabilities, and aLRT measures reflect the probability that a deduced phylogenetic clade is present in a known phylogeny. The authors simulated the evolution of bacterial genes of varying lengths under biologically realistic conditions, and reconstructed those known phylogenies using both maximum likelihood and Bayesian methods. Then, they measured how frequently clades in the reconstructed trees exhibiting particular bootstrap percentages, aLRT values, or posterior probabilities were found in the true trees. The authors have observed that none of these values correlate with the probability that a given clade is present in the known phylogeny. The major conclusion is that none of the measures provide any information about the likelihood that an individual clade actually exists. It is also found that the mean of all clade support values on a tree closely reflects the average proportion of all clades that have been assigned correctly, and is thus a good representation of the overall accuracy of a phylogenetic tree.

## Author Summary

The construction of phylogenetic trees, which depict past relationships between groups of DNA or protein sequences, has valuable application in many fields of study, most commonly evolutionary and population biology. Before drawing conclusions from phylogenetic trees, it is important to assess how accurate those reconstructions are. This is typically accomplished by examining measures of “clade credibility” (such as bootstrap or posterior probability values), which represent how reproducible relationships are within the tree based on the parameters of the phylogenetic analysis. However, such measures do not necessarily reflect how likely inferred relationships are to have actually occurred in nature. Therefore, using simulated data where relationships are known, we have determined how well several measures of clade credibility correlate with the likelihood that a deduced phylogenetic grouping actually exists in reality. Surprisingly, we found no such correlation, and that the inferred relationships were correctly assigned about as often in cases where clade credibility values were very low as where they were high. This finding suggests that current measures of phylogenetic tree reliability are not useful in predicting whether specific inferred relationships have actually occurred.

RETRACTED

## Introduction

Phylogenetic analysis, once the province of systematists and evolutionary biologists, has become a fundamental tool of computational biology and biological disciplines as diverse as biochemistry, epidemiology, and developmental biology. While systematists use phylogenetic analysis of molecular sequences to elucidate the historical relationships among species, other disciplines tend to focus more on the historical relationships of the sequences themselves. The results of phylogenetic analyses are typically presented as phylogenetic trees, diagrams that graphically illustrate those historical relationships. Phylogenetic trees are just estimates of those historical relationships, and it is therefore important to have some way to evaluate the quality and reliability of phylogenetic reconstructions.

The most widely used method of estimating the reliability of trees is the nonparametric bootstrap [1]. The bootstrap method addresses the reliability of the tree topology (the branching order) by calculating the bootstrap percentage (BP) for each interior node, or clade, in a tree. In the bootstrap method, the sites in a set of aligned sequences are randomly sampled with replacement to create a pseudo-alignment, and that pseudo-alignment is used to produce an estimated “bootstrap tree.” Typically, 100–2,000 bootstrap trees are estimated, and the BP for a clade on the original phylogenetic tree is the percentage of the bootstrap trees that also include that clade. Thus, confidence in the groupings of taxa can be estimated. A drawback to the bootstrap method is that it can potentially be very time-consuming. For example, maximum likelihood is at present the most widely used statistical phylogenetic method, but because it is computationally intensive, performing a bootstrap analysis on maximum likelihood trees can require prohibitive amounts of time.

Recently, a new approach to estimating branch (or clade) support, the approximate likelihood ratio test (aLRT), has been introduced [2]. The aLRT is a fast and accurate method for assessing branch support for maximum likelihood trees. Under conventional LRT, the null hypothesis is that the branch has a length of zero (i.e., it does not exist), and the test statistic is 2(*l_1_* − *l_0_*)*,* where *l_1_* is the likelihood of the most likely tree and *l_0_* is the likelihood of the tree in which the branch does not exist. In aLRT, the test statistic is approximated by 2(*l_1_* − *l_2_*), where *l_2_* is the likelihood of the second most likely tree, an approximation that enormously decreases computational time and results in a practical and slightly conservative test statistic. The significance of the aLRT test statistic is calculated from a mixed χ^2^ distribution, with half drawn from zero and half drawn from one degree of freedom. The aLRT approach is implemented in the beta version of PHYML 2.4.5 [3] (http://atgc.lirmm.fr/alrt). The most recent release of the beta version of PHYML also implements an alternative nonparametric Shimodaira–Hasegawa-like (SH-like) procedure that is typically more conservative than the χ^2^ approach, so PHYML now offers the option of assigning support as the smaller of the values calculated by the two methods.

RETRACTED

In the last decade, a new method of estimating phylogenetic trees, the Bayesian method, has gained increasing popularity [4–7]. The Bayesian method, as implemented by the program MrBayes [8,9], estimates the posterior probabilities (PPs) of clades by calculating, among the trees with the highest posterior probabilities, the fraction of the time that each clade appears as those trees are visited in proportion to their probabilities. The Bayesian method has the advantage that it calculates PPs during the process of estimating the consensus tree. It is therefore much faster to obtain PP estimates of clade reliability by the Bayesian method than to obtain BPs of clade reliability by maximum likelihood.

BP, aLRT, and PP are measures of clade support, but they are often presented as measures of the accuracy of the tree [5,10]. None, however, is a metric of accuracy. aLRT assesses the likelihood that a branch exists on a maximum likelihood tree. BP and PP are simply measures of repeatability; BP measures the repeatability with which a clade occurs among subsamples of the data used to create the original tree, and PP measures the repeatability with which a clade occurs among the set of nearly equally likely trees after the Bayesian process has converged on a set of trees with nearly identical likelihoods. Because of discrepancies between Bayesian posterior probabilities and bootstrapped maximum likelihood percentages, there has been considerable controversy about BP versus PP as measures of clade reliability [11–15].

RETRACTED

For real, empirical data, we cannot know the accuracy of a tree because we have no way of knowing the true branching order of the taxa or sequences that are being considered. Simulated datasets, in which the true tree is known, have been used to compare BP and PP with the accuracies of estimated trees. Several such studies have shown that BP underestimates clade reliability (i.e., clades in the estimated tree are more likely to exist in the true tree than is indicated by BP) [10,11,13–16]. There have been conflicting reports about the relationship between PP and accuracy. In general, PP has been found to be less conservative than BP. Some studies [11,12] have concluded that PP is too liberal (i.e., overestimates accuracy), while others [13,14] conclude that PP better reflects accuracy. Another study concluded that BP and PP can be taken as potential upper and lower estimates of accuracy, but that they are not interchangeable and cannot be directly compared [15]. Similarly, Anisimova and Gascuel reported that aLRT using the χ^2^ approach is similar to posterior probabilities, and their unpublished data suggest that the SH-like approach is more conservative than the χ^2^ approach (http://atgc.lirmm.fr/alrt).

The conclusions of the above studies are only as reliable as the extent to which the simulations mimic real evolutionary processes that generate the empirical data to which we actually apply phylogenetic methods. In all cases, the simulations incorporate specific evolutionary models, the most common being the K2P model [17], to guide the simulation process. The results will be no more realistic than the assumptions and biases of that model. Modeling evolution as a process of substitution confounds two distinct processes, mutation and selection, the outcome of which is the real substitution process [18]. The number of taxa used in the simulations reported in [10–16] ranges from four to 28. Many, and probably most, phylogenetic studies involve many more taxa. Typically, branch lengths are uniform, although some studies included a specific pattern of length variation. Importantly, the simulations only consider base substitutions, not insertions or deletions (indels). The resulting sequences thus need not be aligned. In reality, historical indels necessitate using multiple alignment programs to estimate the homologous characters within. The alignment process strongly affects the reliability of the resulting trees. For coding sequences, the accuracy of a tree is significantly increased by aligning the corresponding protein sequences and using that alignment to place the corresponding gaps into the DNA coding sequences [18]. However, when the average percentage identity of the amino acids is within the “twilight zone” of 20%–30%, only 80% of residues are correctly aligned [19], and when identity is below 10%, less than 50% of residues are correctly aligned [20]. The failure to include indels in the simulation process therefore reduces considerably the confidence we can place in applying conclusions drawn from those simulations to real data.

RETRACTED

The EvolveAGene simulation program [18,21] was designed to mimic the evolution of sequences in a more biologically realistic fashion. A real sequence is used for the root node of the tree, and a strictly bifurcating bilaterally symmetrical tree is evolved. Branch lengths are randomly varied from zero to a value chosen by the user. Mutation and selection are treated as separate processes. The mutation process is simulated by introducing random mutations, including base substitutions, insertions, and deletions, into the sequences according to the spontaneous mutation spectrum of *Escherichia coli.* (The mutational spectrum is the experimentally determined relative frequencies with which the various base substitutions and indels of different lengths occur, before selection or drift act on those mutations.) The selection process is simulated by (1) assuming that all frameshift and nonsense mutations are strongly deleterious and thus not accepting those mutations, and (2) accepting nonsynonymous base substitutions with a probability that corresponds to a user-specified nonsynonymous substitution per nonsynonymous site to synonymous substitution per synonymous site (dN/dS) ratio, which can be set to biologically realistic values. The EvolveAGene program has been used to compare accuracies of various phylogenetic methods [18] and to explore the accuracies with which parsimony and Bayesian methods can reconstruct ancestral protein sequences [21].

In this study we are not particularly interested in comparing PP, BP, and aLRT per se. Instead, we are interested in asking two questions: (1) for all measures of clade credibility, how well does the credibility of a clade reflect the probability that that clade really exists on the true tree; and (2) how well does the average clade support reflect the topological accuracy of the tree? Topological accuracy is defined as the fraction of clades on the estimated tree that actually exist on the true tree. In this study, both the true tree and the estimated trees are strictly bifurcating, so the number of interior clades is the same. Thus, the number of false positive errors (clades found on the estimated tree that do not exist on the true tree) is identical to the number of false negative errors (clades on the true tree that are not on the estimated tree). We simulate the evolution of several genes under biologically realistic conditions and find that none of the estimates of clade support correlates with topological accuracy; in other words, clade supports tell us nothing about the likelihood that an inferred clade actually exists. However, we find that the average clade support does correlate well with the topological accuracy of the tree.

RETRACTED

## Results/Discussion

Ten simulations were initiated from each of five E. coli K12 coding sequences to assess how well BPs from maximum likelihood trees, aLRT support by the χ^2^ approach, aLRT support by the minimum of SH-like and χ^2^ approaches, and posterior probabilities from Bayesian trees corresponded to clade accuracies. The simulation conditions were chosen to generate datasets that were at the practical limits for reliable alignments. Indeed, the typical average Jukes–Cantor [22] distances among the sequences for those datasets was 1.39 ± .02 substitutions per site, well above the limit of 1.0, above which Nei and Kumar [23] state that neighbor-joining trees are unreliable.

We define “true clades” as clades in the estimated tree that exist in the true tree, and we define “accuracy” as the percent of the total clades in the estimated tree that are true clades. Tables 1–4 show, respectively, the results for Bayesian trees and for maximum likelihood trees by the bootstrap and the two aLRT approaches. In each case, rows are ranges of clade credibility values.

**Table 1:** Bayesian Trees

**Table 2:** Maximum Likelihood Tree Bootstrap Clade Support

**Table 3:** Maximum Likelihood Tree aLRT Clade Support by χ^2^ Test of Significance

**Table 4:** Maximum Likelihood Trees aLRT Clade Support by Minimum of SH-Like and χ^2^ Test of Significance

For all methods, accuracy increases as the lengths of the sequences increase. Mean BPs are conservative estimates of mean topological accuracy, and in keeping with [13] and [14] we find that average posterior probabilities are a better estimate of topological accuracy than are BPs. BPs underestimate accuracy, particularly for trees based on the shorter sequences, more than do posterior probabilities or aLRT supports. We do not interpret this finding to mean that BPs should be the “gold standard” measure of reliability; indeed, we find the notion that the less-accurate estimate should be the gold standard to be slightly ludicrous.

Our results, however, differ strikingly from those of [13] and [14] with respect to the correspondence between individual clade confidences and the accuracy of those clades. Alfaro et al. [13] found that for most topologies accuracy was higher than either BP or PP when clade confidences were greater than ∼40%, but lower than clade confidences when those measures were less than ∼40%. Hillis and Bull [10] obtained similar results for BP, and Wilcox et al. [14] obtained similar results for PP, but a low crossover point at about 20% for BP. In contrast, we find no significant correlation between individual clade supports and the probability that a clade is correct, whichever method of clade support is used. We regressed the fraction of clades that actually exist within each decile against the midpoint for each decile of clade support; thus, a slope approaching one would be expected for a perfect correlation between those values, whereas a slope of zero would indicate no correlation. Only two out of the 28 plots have slopes that are significantly different from zero (genes *nuoK* and *rplF* for bootstrap support of maximum likelihood trees, with *p* = 0.03 and 0.02, respectively). One of these slopes is slightly positive, and the other is slightly negative; thus, both likely represent outliers.

RETRACTED

The absence of correlation between clade support and the likelihood that a clade exists means that, whatever the method, clade support values provide no information about, and have no predictive power as to, the likelihood that the clade exists. We attribute the differences between our results and those of others [10,13,14] to our use of a more biologically realistic simulation.

It is conceivable that this startling finding is the result of reconstructing relatively large (64 taxon) trees under some false assumption that is unknowingly incorporated into the simulation: perhaps with so many taxa, resulting in an enormous number of possible trees, any clade that has even mild support is likely to be a true clade. We think this possibility is unlikely, because the fraction of false clades that have 81%–100% support is roughly the same as the fraction of false clades that have low (0%–40%) support. Nevertheless, to test the idea that our findings are an artifact of considering large trees, we tested all four methods with 16-taxon datasets of *nuoK,* replicated ten times each. (The *nuoK* gene was chosen because it is the shortest gene and the gene for which all methods were the least accurate.) As before, the taxa were a random sample from a 128-taxon dataset. When the number of taxa was reduced from 64 to 16, the quality of the alignments was reduced so that the amino acid identity was <20%, below the zone in which alignments are reliable. The average branch length was therefore reduced from 0.18 to 0.15 substitutions per site to produce alignments that exhibited an average of 24% amino acid identity, well within the “twilight zone” [19]. Table 5 shows that the results are essentially the same as in Tables 1–4: there is no significant correlation between clade support and the fraction of true clades. Both mean accuracy and mean clade support are generally lower than in Tables 1–4, but it remains the case that clade support provides no information about the likelihood that a clade actually exists.

RETRACTED

**Table 5:** *nuoK* (300 bp) Trees Based on 16 Random Sequences Sampled from 128 Evolved Sequences

Random sampling of taxa typically results in well-balanced trees (Figure 1), and it is conceivable that our findings apply only to trees with similar topology. To test that possibility, we nonrandomly sampled ten *nuoK* datasets to generate highly pectinate, unbalanced 16-taxon trees (Figure 2). For the unbalanced trees, the topological accuracies were higher than for the 16-taxon balanced trees, and all methods of clade support again underestimated that accuracy. Again, there was no significant correlation between clade support and the likelihood that a clade existed on the true tree (Table 6).

**Figure 1:** Typical Phylogenetic Trees (A) True 64-taxon tree initiated with *nuoK* sequences. The arrow indicates a near trichotomy. (B) Bayesian tree estimated from the same data as in (A). Numbers are posterior probabilities of clades whose posterior probabilities are <90%. Arrows indicate the clades that do not exist in the true tree.

**Figure 2:** Topology of a Typical Unbalanced Tree of 16 Taxa

**Table 6:** *nuoK* (300 bp) Unbalanced Trees Based on 16 Sequences Sampled from 128 Evolved Sequences

We conclude that our results are general, and not simply attributable to large trees or to balanced trees.

This is one of those good news–bad news stories beloved by comedians. The bad news is that none of the methods of assessing clade support provides any reliable estimation that the clade has been correctly assigned. The good news is that, even with data that are near the practical limits for phylogenetic tree reconstruction, both maximum likelihood and the Bayesian method estimate topologies so well that even when clade support is very low there is a better than 80% chance that the clade is correctly assigned.

In addition, for each method, averaged over the 70 datasets, there is a significant correlation between the average branch support and the accuracy of the tree (Table 7), and for all methods except nonparametric bootstrap, the average clade support value is a good, if slightly conservative, estimator of the overall fraction of clades that actually exist. It might be argued that having a good estimate of overall accuracy is not very useful, and that we are generally interested in identifying unreliable branches. Our results show that we simply cannot identify what particular branches are unreliable based on measures of clade support. Thus, with current methods of determining clade credibility we cannot have what we might generally want, and it is important to acknowledge the limitations of those metrics. On the other hand, methods of determining clade confidence do provide a good estimation of the overall reliability of a phylogenetic tree, and permit us to infer how many untrustworthy branches may be present. Just as we can make good predictions about the diffusion of a mass of molecules over time, but not about the motions of individual molecules in that mass, we can make good estimations of the overall topological accuracy of a tree, but not about the accuracy of individual branches.

RETRACTED

**Table 7:** Mean Clade Support versus Mean Accuracy

## Materials and Methods

### Simulations.

Simulations were performed by EvolveAGene [18,21]. Five coding sequences from E. coli K12 were selected from the E. coli genome entirely on the basis of length, and used to initiate the simulations: *nuoK,* 300 bp, encodes the NADH dehydrogenase subunit K; *rplF,* 530 bp, encodes 50S ribosomal protein L6; *tauB,* 763 bp, encodes a taurine transport ATP-binding protein; *add,* 999 bp, encodes adenosine deaminase; and *araB,* 1,698 bp, encodes ribulokinase. The genes are not functionally related to each other, and none exhibits detectable homology to another by pairwise BLAST comparisons. For the simulations in Tables 1–4, the average branch length was 0.18 substitutions per site, with lengths ranging from 0 to 0.36 substitutions per site; for Tables 5 and 6 the average branch length was 0.15 substitutions per site, ranging from 0 to 0.30 substitutions per site. The tree was evolved for seven “generations” to give 128 terminal taxa; thus, the average length from the root to the tip was 1.26 substitutions per site. The probability of accepting an indel was 0.02, and the probability of accepting a nonsynonymous base substitution was 0.2. Ten independent simulations were carried out from each of the five root sequences.

When all of the terminal sequences descended from the root node were included in the dataset, both Bayesian and maximum likelihood trees included very few nodes with clade confidences <80% (unpublished data). When trees were based on a random subsample of the sequences, both methods produced trees with more low-confidence clades. Datasets used to estimate trees were therefore based on a random sample of 16 or 64 of the 128 evolved sequences.

RETRACTED

### Alignments.

Sequences were aligned by ClustalW [24] as implemented by MEGA 3.1 [25]. Sequences were translated to their corresponding protein sequences by MEGA 3.1, aligned with a gap-opening penalty of 3.0 and a gap-extension penalty of 1.8. The average pairwise amino acid identities in the resulting alignment were typically 21%–22%, near the lower boundary of the “twilight zone” below which alignments are not sufficiently reliable to produce valid phylogenetic trees [19,20]. Triplet gaps corresponding to the gaps in the protein alignment were introduced back into the DNA sequences by MEGA 3.1. The resulting DNA sequence alignments were saved in the FASTA format and converted to the PHYLIP format (for input to PHYML) and to the Nexus format (for input to MrBayes) by a Perl script.

### Estimation of phylogenetic trees.

Trees were estimated by two methods: maximum likelihood as implemented by PHYML 2.4.4 [3], and the Bayesian method as implemented by MrBayes 3.1.2 [9]. In both cases, trees were estimated using the GTR + invariants + gamma model.

For maximum likelihood trees, clade confidences were estimated from 100 bootstrap replicates.

Bayesian trees were estimated from 600,000 generations, sampling every 100 generations, with a heating parameter of 0.15, in two parallel runs. The consensus trees were calculated using the allcompat option (strict consensus) from the final 4,501 trees of each run. Convergence, as judged by the diagnostic average standard deviation of the split frequencies between two parallel runs falling below 0.02, typically occurred before generation 120,000 (1,200 trees).

A typical true tree, in this case initiated with the *nuoK* sequence, is shown in Figure 1A. Note that the true tree includes one near trichotomy, and that the distance from the root to the tips ranges from 0.52 substitutions per site for taxon ZZZZZZZ to 1.55 substitutions per site for taxon PPPPPPPPPP. The corresponding Bayesian estimated tree is shown in Figure 2. Posterior probabilities <90% are indicated. This Bayesian tree is typical in that only 12 of the 61 interior nodes have posterior probabilities <90%, but only four of those low-PP clades (indicated by arrows) are not present in the true tree.

### Calculation of topological accuracy.

A Perl script, InferAcc, was used to compare the estimated trees with the true trees. Clades were sorted into bins as indicated in Tables 1–6, and the clade was scored as existing if it was present in the true tree. Mean accuracy is the fraction of clades in the estimated tree that exist in the true tree averaged over the ten trees in the set.

## Abbreviations

aLRT: approximate likelihood ratio test
BP: bootstrap percentage
indels: insertions or deletions
PP: posterior probability
SH-like: Shimodaira–Hasegawa-like
